# Artificial Intelligence-Based Spiral CT 3D Reconstruction in Transcatheter Aortic Valve Implantation

**DOI:** 10.1155/2022/5794681

**Published:** 2022-05-04

**Authors:** Kunpeng Zhang, Yan Gao, Junwei Lv, Jian Li, Jingli Liu

**Affiliations:** ^1^Department of Catheterization Room, The Affiliated Yantai Yuhuangding Hospital of Qingdao University, Yantai, 264000 Shandong, China; ^2^Department of Computer Tomography Room, The Affiliated Yantai Yuhuangding Hospital of Qingdao University, Yantai, 264000 Shandong, China

## Abstract

To evaluate the clinical application effect of spiral computed tomography (CT) three-dimensional (3D) reconstruction based on artificial intelligence in transcatheter aortic valve implantation (TAVI), a CT 3D reconstruction model based on deep convolutional neural networks (DCNN) was established in this research, which was compared with the model-based iterative reconstruction (MBIR) and used in clinical practice. Then, 62 patients with aortic stenosis (AS) who underwent TAVI surgery were recruited as the research objects. The accuracy, sensitivity, and specificity of the multislice spiral CT scan (MSCT) and transthoracic echocardiography (TTE) in predicting the type of TAVI surgical valve were compared and analyzed. The results showed that the mean absolute error (MAE) (0.01) and root mean square error (RMSE) (0.086) of the MBIR model were higher than the reconstruction model in this research. The structural similarity (SSIM) (0.831) and peak signal-to noise ratio (PSNR) (32.77 dB) of the MBIR model were lower than the reconstruction model, and the differences were considerable (*P* < 0.05). Of the valve models selected based on the TTE measurement results, 35 cases were accurately predicted and 27 cases were incorrectly predicted. The accuracy of MSCT was 87.1%, the specificity was 98.84%, and the sensitivity was 92.87%; all of which were significantly higher than TTE (*P* < 0.05). In summary, compared with the MBIR reconstruction model, the imaging results of the model established in this research were closer to the real image. Compared with TTE, MSCT had higher accuracy, sensitivity, and specificity and can provide more accurate preoperative predictions for patients undergoing TAVI surgery.

## 1. Introduction

Aortic stenosis (AS) is a common valve disease and its incidence increases with age. Some studies have shown that the incidence rate in people over 75 years old is about 5% [1, 2]. The clinical manifestations of AS are chest tightness, dyspnea, and even myocardial infarction and sudden death in patients with inflammation [3]. AS can lead to increased pressure load of the left ventricle, resulting in a shortened diastolic period and prolonged ejection time [4]. The pathogenic causes of AS include inflammation, degenerative changes, and congenital developmental malformations. The most common lesions of AS abroad are degenerative calcification in old age, while the most common cause of AS in China is rheumatic heart disease [5–7].

Surgical aortic valve replacement (SAVR) is the first choice for patients with severe AS [8–10]. However, since most patients with AS are elderly people over 70 years old, they are often accompanied by diseases such as renal failure and chronic obstructive pulmonary disease, which greatly increase the risk of surgery [11, 12]. Transcatheter aortic valve implantation (TAVI) is one of the hot topics in cardiovascular research in recent years. Compared with SAVR, this technique has less trauma, lower risk, and fewer contraindications and is suitable for AS patients who cannot be treated with SAVR [13, 14]. The operation path of TAVI mainly includes the anterograde method and the method of operation. Both of these surgical methods belong to the complicated interventional treatments, which have strict requirements for imaging examinations, requiring high accuracy and clear imaging [15]. At present, the clinical imaging methods used to assess AS mainly include transthoracic echocardiography (TTE), nuclear magnetic resonance (MRI), and multislice spiral CT scan (MSCT) [16, 17]. Echocardiography is a noninvasive examination, and there is no radiation damage. The operation is simple, but the imaging quality is not good, and it is greatly affected by the operation level of the clinician [18]. Cardiac MRI is not affected by the gas in the bones and lungs, and clearly shows the internal conditions of the heart. The imaging results have better spatial and temporal resolution and are less affected by the level of the operator. However, the technology has many contraindications, and the cooperation of the examinee is required [19]. MSCT combines the advantages of ultrasound and MRI technology, can clearly show the structure and spatial relationship of normal tissue and lesion tissue, and is widely used in assessing the degree of calcification and valve stenosis in AS patients [20, 21].

However, traditional CT imaging is based on a large amount of projection data, which increases the reconstruction time while also increasing the radiation dose received by the patient [22]. Therefore, how to reduce the number of scans and reduce the radiation dose has become a hot topic for many scholars [23]. Some scholars used intelligent algorithms to train image segmentation models in a large number of datasets, which speeds up imaging and improves imaging quality [24]. Among them, deep learning is the most widely used. Kong et al. [25] used the volume neural network to achieve the segmentation of CT images, and the effect was good. However, the establishment of the model is based on a huge dataset. If the data of each patient is trained, it will greatly increase the training time and reduce the imaging efficiency [26].

Based on the abovementioned factors, TAVI is one of the hot topics in cardiovascular research in recent years and MSCT can accurately reflect the structure and spatial relationship of the tissues around the lesion. The neural network can effectively improve the imaging quality. Therefore, the deep convolutional neural network (DCNN) was employed in this research to perform CT 3D reconstruction and to evaluate the application of TAVI in AS treatment and prognostic analysis. This research is aimed at providing a reliable treatment method for AS patients and reducing mortality and improving the quality of life of patients.

## 2. Materials and Methods

### 2.1. Research Objects

A total of 62 patients with AS in the hospital from February 2019 to June 2020 were selected as the research objects. There were 38 males and 24 females, aged from 49 to 80 years, with an average age of 70.23 ± 5.3 years. All patients underwent preoperative MSCT and TTE examination. This study had been approved by the ethics committee of the hospital. Patients and their families were aware of this research and have signed the informed consent.

Inclusion criteria are as follows: (i) patients with poor compliance in examination, (ii) patients with contraindications for CT examination, and (iii) patients with complete clinical data.

Exclusion criteria are as follows: (i) patients with mental diseases, (ii) patients who dropped out of the experimental group due to personal factors, and (iii) patients who cannot cooperate with the follow-up.

### 2.2. Imaging Methods and Image Analysis

In this research, patients were examined by 64 slice spiral CT. The scanning layer thickness was 625 mm × 64 mm, the rack speed was set to 0.42 s/360°, the tube voltage was set to 120 kV, and the tube current was set to 100–210 mAs. A nonionic iodine pair agent (iopamidol 370 mg I/mL) was used for 52–140 mL, and a contrast agent was used according to the patient's body weight and specific conditions. The injection rate was controlled at 4–5 mL/s. The region of interest was located in the aorta, the trigger threshold was set to 110 HU, and the scanning range was from the tracheal carina to the diaphragmatic surface of the heart. The scanning time was 4.8 to 10 seconds. The reconstruction thickness was set to 0.67 mm, and the data was stored after the scanning was completed. Transthoracic echocardiography was performed using Philips iE33 and the corresponding probe (transthoracic SS-1).

Image processing was implemented by the heart software provided by Excel Brilliance Walkspace (EBW) for image reconstruction and analysis, including volume present (VR), multiplane reconstruction (MPR), surface reconstruction (CPR), and maximum intensity projection (MIP).

### 2.3. DCNN CT 3D Reconstruction Model Establishment

The basis of image reconstruction is that when X-ray irradiates an object, it interacts with the object and then attenuates. The attenuating effect is regarded as the absorption of X-ray by the object, so as to obtain the imaging result of the object (Figure 1). It is set that *N* is the intensity of the incoming X-ray light, *N*_1_ is the intensity of attenuated light after the X-ray passes through the object, *μ* is the attenuation coefficient, *K* is the thickness of the object, and then, the relation between *N* and *N*_1_ is mapped as the following equation.

(1) $$\begin{array}{c} {\text{N}}_{1}=Ne^{-\mu K}. \end{array}$$

In practical application, the thickness of objects is not uniform, for example, the thickness and density of human bones and muscles are inconsistent, so equation (1) does not meet the actual requirements. The object is subdivided into *m* modules, then, there is a thickness *k* in each module, and the attenuation coefficient of the module is denoted as *μ*_1_, *μ*_2_, ⋯, *μ*_*i*_; then, the mapping between *N* and *N*_1_ is redefined as follows.

(2) $$\begin{array}{c} N_{1}=N\exp\left(-k\underset{i=1}{\overset{m}{\Sigma }}\mu_{i}\right). \end{array}$$

To obtain a more accurate reconstruction, as *k* approaches infinitely small, the linear integral is derived from the probe plate to equation (2), as shown as follows.

(3) $$\begin{array}{c} P=\underset{N}{\int \mu }\left(x\right)kx. \end{array}$$

Shen et al. [27] designed a hierarchical neural network and used it in the structured training process of ultrasparse projection view data to complete the prediction of 2D images to 3D images generated by X-ray. The feature space conversion (encoder-decoder) framework was added to 2D imaging and 3D imaging, and the 3D image of the object was successfully obtained from 2D imaging after training. Based on Shen et al.'s work, this work added residual paths of feature images to the generation network to obtain a CT 3D reconstruction model framework (Figure 2).

### 2.4. Observation Indexes

According to the number of aortic valve rings and the shape of the aortic root of the patient, the appropriate valve type was selected. Aortic valve annulus diameter measurement was implemented by the 3D measurement method, which measured the aortic valve annulus diameter, and the attachment point of aortic valve was delineated on the aortic valve. In the reconstructed 3D image, the lowest point of three arched aortic valves was taken out to determine a plane and the long axis diameter and short axis diameter of the plane were measured.

The collected data samples were adjusted uniformly to a 128 × 128 size, and normalized to obtain 2D network data as the input image. Mean absolute error (MAE), root mean square error (RMSE), structural similarity (SSIM), and peak signal-to-noise ratio (PSNR) were calculated to measure the quality of the image reconstruction.

### 2.5. Statistical Treatment

The data processing in this research was analyzed by SPSS 19.0. Measurement data was expressed by the mean plus or minus standard deviation ($\overset{¯}{x}\pm s$), and the count data was expressed by the percentage (%). One-way analysis of variance was used for pairwise comparison. The difference was considerable at *P* < 0.05.

## 3. Results

### 3.1. Model Performance Evaluation

MBIR was introduced and compared with the proposed model regarding the MAE, RMSE, SSIM, and PSNR of the two models. The results were shown in Figure 3. The MAE (0.01) and RMSE (0.086) of the MBIR model were significantly higher than those of the reconstruction model in this research. The SSIM (0.831) and PSNR (32.77 dB) of the MBIR model were significantly lower than those of the reconstruction model in this research, and the differences were substantial (*P* < 0.05). It showed that the imaging result of the reconstruction model in this research was closer to the real image and the image resolution was relatively higher and the imaging effect was good.

MSE of the training sample and the validation sample of cardiac CT was compared during the training process (Figure 4). The proposed model fitted the training data well and had a good effect on the data not included in the training dataset.

### 3.2. Algorithm Reconstruction Result

Figure 5 showed the 3D reconstruction of the cross-sectional images of the heart CT processed by the proposed reconstructed model and MBIR model. The proposed reconstructed model had a better effect, and the reconstructed image was closer to the real image. It further illustrated that deep learning technology has the potential for development in the application of CT 3D reconstruction applications.

### 3.3. Measurement Result of the Aortic Valve Annulus Diameter (MSCT)

A total of 62 patients were included. Among them, 42 patients had tri-leaflet valves and 20 patients had two-leaf valves. The measured annulus diameter of all patients was shown in Figure 6.

### 3.4. TTE Measurement Results and TAVI Surgery Results

Valve models selected by 62 patients after TAVI were counted based on aortic ring diameter measurement results and compared with TTE measurement results (Figure 7). Valve type 23 was used in 4 of 62 patients, while 43 patients were treated with valve type 26. Valve type 29 was used in 13 patients. The valve model 32 was used in 2 patients. According to the results of TAVI operation, 54 cases were predicted accurately according to the results of MSCT measurement and the accuracy was 87.1%. According to the measurement results of TTE, 35 cases were predicted accurately, the accuracy was 56.45%, which was significantly lower than MSCT, and the difference was considerable (*P* < 0.05).

Based on the results of MSCT and TTE (predictive value) and surgical results (true value), the sensitivity and specificity of MSCT were 92.87% and 98.84%, respectively. The sensitivity and specificity of TTE were 82.31% and 49.52%, respectively. Receiver operating characteristic (ROC) curves of TTE and TTE were drawn in Figure 8, and the difference between TTE and TTE was considerable (*P* < 0.05).

## 4. Discussion

AS is a common heart valve disease in the elderly, leading to heart failure risk, high surgical risk, and poor prognosis. The development of TAVI technology provides a new path for patients who cannot be treated with SAVR due to their own complications. Sehatzadeh et al. [28] evaluated the safety, efficacy, and cost effectiveness of TAVI in elderly patients with symptomatic aortic stenosis. The results showed that the one-year mortality of TAVI and SAVR was similar and the survival rate of patients who could not receive SAVR but chose TAVI was significantly improved. In addition, the diameter of the aortic valve ring should be obtained through imaging examination before TAVI treatment and the appropriate valve type should be selected according to the examination results. Inappropriate valve type and size will lead to pathological changes of surrounding annulus and aortic regurgitation, which will seriously affect the prognosis of patients [29, 30]. In this research, a 3D CT reconstruction model based on DCNN was proposed based on artificial intelligence and MBIR reconstruction model was introduced. MAE, RMSE, SSIM, and PSNR of the two models were compared. The results showed that the SSIM and PSNR of the reconstruction model presented in this work were significantly lower than those of MBIR model, while SSIM and PSNR were significantly higher than those of the MBIR model, and the difference was statistically significant (*P* < 0.05). This indicated that the reconstruction model had better performance in CT image processing and the image quality obtained by the reconstruction model was significantly better than that obtained by traditional algorithms.

In this research, the trained model was applied into clinical practice. 62 AS patients were selected as research objects, and the diameter of the aortic valve ring of all patients was measured by MSCT and TTE. According to the measured results, a suitable valve type was selected (the predicted value) and the predicted value was compared with the actual value of the operation. León Del Pino et al. [31] explored the risk factors of prosthesis-patient mismatch (PPM) in 185 patients after TAVI surgery. The results showed that the higher European cardiovascular risk factor score (Euro Score), smaller prosthesis size, and smaller aortic ring diameter were associated with PPM. After TAVI, 4 of 62 patients had valve type 23, while 43 patients were treated with valve type 26. Valve type 29 was used in 13 patients, and valve type 23 was used in 2 patients. The valve type used in TAVI surgery was selected according to the diameter, area, and circumference of the aortic valve ring, and an appropriate valve type was the key to successful surgery [32]. In this research, 54 cases of valve models selected based on MSCT measurement results were correctly predicted, while 8 cases were incorrectly predicted. Among the valve models selected according to TTE measurement results, 35 cases were correctly predicted and 27 cases were incorrectly predicted. The accuracy, sensitivity, and specificity of the two methods were compared based on TAVI results. The results showed that the accuracy, specificity, and sensitivity of MSCT were 87.1%, 98.84%, and 92.87%, respectively, which were significantly higher than those of TTE (*P* < 0.05). Preoperative evaluation of TTE can measure the internal anatomical structure and valve size of the heart in real time, but it is easily affected by the operator level and aortic valve calcification, so the measurement results of TTE are small. Doris et al. [33] evaluated the severity of aortic stenosis in patients with aortic valve calcification by CT quantification (CT-AVC) and conducted a comparative study with echocardiography. The results showed that CT-AVC was reproducible and the measurement reproducibility became more standardized over time, with higher accuracy than echocardiography, which was similar to the results of this research.

## 5. Conclusion

The DCNN-based CT 3D reconstruction model was established in this research based on artificial intelligence technology, and the MBIR reconstruction model was introduced and applied in clinical practice. The accuracy, sensitivity, and specificity of MSCT and TTE in predicting valve types after TAVI surgery were compared and analyzed in 62 AS patients who underwent TAVI surgery. The results showed that compared with the MBIR reconstruction model, the imaging results of the model established in this research were closer to the real image and the image quality was better. Compared with TTE, MSCT had higher accuracy, sensitivity, and specificity and can provide more accurate preoperative prediction for patients undergoing TAVI surgery. However, there is a lack of research on the prognosis of TAVI patients in this research. Moreover, due to the limitation of the sample size, it is difficult to carry out a multicenter study, so further discussion on clinical application is needed in the follow-up study. Overall, this research provides a new approach for the selection of valve types for AS patients undergoing TAVI surgery.

## Figures and Tables

**Figure 1:** Schematic diagram of X-ray attenuation.

**Figure 2:** CT 3D reconstruction model framework.

**Figure 3:** Model performance evaluation. (a) Showed the MAE and RMSE; (b) showed the SSIM and PSNR. ∗ indicated that the difference was significant compared to the reconstruction model in this research (*P* < 0.05).

**Figure 4:** Heart CT loss curve.

**Figure 5:** 3D reconstruction of the cross-sectional CT image of the heart. (a) Showed the real image; (b) showed the image processed by the reconstruction model proposed; (c) showed the image processed by the MBIR model.

**Figure 6:** Measurement results of the aortic valve annulus diameter.

**Figure 7:** Comparison of MSCT and TTE measurement results. (a) Showed the TAVI operation results; (b) showed the comparison of MSCT and TTE measurement results. ∗ indicated that TTE was considerable compared to MSCT (*P* < 0.05).

**Figure 8:** ROC curve for predicting the accuracy of valve models. (a) MSCT; (b) TTE.

## Data Availability

The data used to support the findings of this study are available from the corresponding author upon request.
